# Small Intestinal Tumors: A Rare Case of Tubulovillous Adenoma in Duodenum

**DOI:** 10.7759/cureus.4671

**Published:** 2019-05-15

**Authors:** Mustafa N Malik, Zunairah Shah, Abdul Rafae, Tayyab Mahmood, Hafiz M Fazeel

**Affiliations:** 1 Internal Medicine, The University of Arizona, Tucson, USA; 2 Hematology and Oncology, The University of Arizona, Tucson, USA; 3 Internal Medicine, McLaren Flint - Michigan State University, Flint, USA; 4 Internal Medicine, Federal Government Services Hospital, Rawalpindi, PAK

**Keywords:** small intestinal tumors, small intestinal tumors, duodenal tumors, duodenal tumors, tubulovillous adenoma, villous adenoma, tubulovillous adenoma, villous adenoma, familial adenomatous polyposis, familial adenomatous polyposis

## Abstract

The small intestine is a relatively privileged organ; primary tumors are uncommon among malignancies of the gastrointestinal tract, with an average annual incidence rate of 9.9 per million people. Among these uncommon tumors, duodenal tumors are even rarer with an average incidence rate of 0.4% only. Histopathological examination mostly shows villous type. Tubulovillous histology is extremely rare with an incidence of less than 1% of all duodenal tumors. These tumors are either found incidentally or during screening for familial disorders such as familial adenomatous polyposis or Gardner’s syndrome. Patients usually have symptoms such as diarrhea and abdominal pain along with weight loss over a period of months. Itching over the whole body and progressive yellow discoloration of sclera and skin (jaundice) can also be present when tumor compresses the common bile duct (CBD) and causes obstruction, especially in the region of ampulla of Vater. Examination of the abdomen may or may not reveal a mass lesion. Abdominal radiography and ultrasound show intra- and extra-hepatic biliary dilatation along with distention of CBD and growth at the lower end of CBD. Endoscopic retrograde cholangiopancreatography (ERCP) is, however, the investigation of choice as it not only allows direct visualization of a biliary tree but biopsy specimens can also be taken. Palliative procedures like placing a stent in the common bile duct to relieve obstruction can be done or a drain can be placed to drain bile. The definitive treatment is the Whipple procedure involving gastrojejunostomy, choledochojejunostomy, and cholecystectomy. Our case is unique as the patient had duodenal tubulovillous adenoma, a very rare tumor among the already uncommon duodenal tumors. The patient underwent Whipple procedure, T tube was placed, and feeding jejunostomy was done. An uneventful recovery occurred.

## Introduction

Small intestinal primary tumors are quite rare with an incidence equal to one-tenth of the similar tumors of the colon [1]. Less than 1% of all duodenal neoplasms comprise tubulovillous adenomas. Approximately 88% of all the tubulovillous adenomas are found in the second part of the duodenum, while the rest 12% are found in the first and third part of the duodenum with equal distribution in both [2-3]. These tumors arise either sporadically or as a part of certain genetic syndromes such as Gardner’s syndrome, familial adenomatous polyposis (FAP) [4-5]. These tumors tend to cause bleeding or intestinal obstructions commonly at the duodenum and ampulla of Vater. They are usually found incidentally during upper gastrointestinal endoscopy, familial adenomatous polyposis surveillance, and evaluation of symptomatic ductal obstruction. Tumors of the ampullary region have a tendency to malignant transformation with approximately 15% to 25% of the lesions develop into malignant neoplasms. This rate is even higher once the tumor size exceeds two centimeters (cm). It is, therefore, important to act vigilantly when dealing with these tumors and perform a biopsy with resection and watchful follow-up of these lesions [6]. We report a unique case of a 64-year-old female who presented with painless progressive jaundice and weight loss due to periampullary tubulovillous adenomas of the duodenum.

## Case presentation

A 64-year-old female presented to the outpatient clinic with a four-month history of painless progressive jaundice of skin and eyes along with loss of appetite and weight loss. On further inquiry, patient-reported one-month history of generalized itching was gradual in onset, intense at times, and mostly involved hands, forearms, and abdomen. There was also a history of pale stools and dark urine along with on and off melena. On review of systems, the patient denied abdominal pain, fever, epigastric discomfort, nausea, hematemesis, vomiting, constipation, or diarrhea. Family history was negative for any familial pathologies such as familial adenomatous polyposis or colorectal carcinoma in first degree relatives. Physical examination revealed a 4 x 2-cm reducible swelling in the epigastric region upon palpation. The abdomen was soft and non-tender otherwise.

Laboratory investigations showed elevated total serum bilirubin level (17.5 mg/dl), alkaline phosphatase (ALP; 1356 IU/L), and alanine aminotransferase (ALT; 315 IU/L). Other laboratory parameters including serum electrolytes, serum amylase, serum lipase, and coagulation profile were observed to be normal. Abdominal ultrasonogram showed dilated intra-hepatic biliary channels, distended gall bladder with the normal appearing pancreas. Common bile duct (CBD) was distended up to 2.1 cm with a 1.8 x 1.4 cm growth at its distal end (Figure 1).

**Figure 1:** Abdominal USG showing dilated common bile duct with growth at the distal end USG, ultrasonogram

Computerized tomography (CT) scan of the abdomen confirmed moderate dilatation of intra & extrahepatic biliary channels and dilated CBD up to its lower end (Figure 2).

**Figure 2:** Dilated CBD on abdominal CT scan CBD, common bile duct; CT, computed tomography

Endoscopic retrograde cholangiopancreatography (ERCP) along with biopsy was scheduled and a double pigtail plastic stent (10 x 5 cm) was placed at the ampulla to achieve free drainage of the bile. Results of ERCP-guided biopsy showed papillary formation lined by cells showing mild atypia (Figure 3).

**Figure 3:** ERCP biopsy specimen showing tubulovillous adenoma of the duodenum ERCP, endoscopic retrograde cholangiopancreatography

The diagnosis of tubulovillous adenoma of the duodenum was made, and Whipple procedure (gastrojejunostomy, pancreaticoduodenectomy, pancreaticojejunostomy, choledochojejunostomy, and cholecystectomy) was done along with T-tube placement and feeding jejunostomy (Figure 4).

**Figure 4:** Intra-operative view of duodenal tubulovillous adenoma

No postoperative complications were observed and the patient was discharged on the eleventh postoperative day. T-tube was removed 10 days after discharge and a follow-up cholangiogram was done which came out to be normal.

## Discussion

The small intestine is the longest part of the gastrointestinal tract, accounting for 75% of its length and 90% of the mucosal surface. Of all the gastrointestinal malignancies, benign tumors are approximately 3% to 6%, while malignant tumors are 1% to 3% [7]. Small bowel tumors include carcinoids, adenocarcinomas, lymphomas, sarcomas, gastrointestinal stromal tumors as well as a variety of benign polyps [8]. Over forty different histological subtypes of malignant tumors have been identified but the four most common include adenocarcinoma, neuroendocrine tumors, sarcomas and lymphomas [9]. Benign lesions include polyps such as found in familial adenomatous polyposis (multiple small bowel polyps), Peutz-Jeghers syndrome (benign hamartomatous polyps) and Gardner’s syndrome [10].

Adenomas are commonly found tumors of the colon. However, they can also occur in the upper part of intestine especially in the duodenum with an overall incidence of 0.4% of the lesions found during endoscopic studies [11- 12]. The duodenal villous tumor was first described by Perry in 1893 and was named as duodenal papilloma. Tubulovillous tumors of the duodenum are very uncommon comprising of less than one percent of all duodenal neoplasms [13]. Komorowski et al. in his review of surgical and autopsy material collected over 30 years reported only eight villous tumors of the duodenum [2]. These tumors are named according to the tumor stage as well as its morphology, i.e., villous adenoma, papillary adenoma, villous papilloma, tubulovillous adenoma, and villoglandular polyp [11].

Tubulovillous adenomas may include small, sessile, or polypoid lesions. They are discovered incidentally on endoscopy. Duodenal villous and tubulovillous tumors are often clinically silent [13]. Though they are mostly asymptomatic, sometimes they may present with the signs and symptoms of jaundice (obstructive jaundice), abdominal pain, melena, hematochezia, fever, malaise or weight loss. Physical examination may reveal hard epigastric areas on palpation. Imaging can reveal an ulcerated tumor, dilatation or extensive involvement of the common bile duct and/or pancreatic duct [1]. These tumors can also present with some serious complications such as pancreatitis, duodenal obstruction or intussusceptions [14-15]. The diagnostic test of choice is endoscopy with biopsy of the mass, usually around the ampulla of Vater. Tubulovillous adenomas show a combination of tubular and villous architecture (villous component greater than 25%) and are usually intramural with intraepithelial tumor cells [16].

The treatment technique is usually decided on the basis of size, extent, and location of the tumor as well as its histopathology [11]. These tumors are usually treated surgically using different techniques including polypectomy, duodenotomy, duodenal segment resection, and submucosal excision or duodenopancreatectomy [17]. Recurrence of benign villous tumors after local excision is common and may be malignant. Among patients with adenomas of the duodenum who had a local excision on endoscopic surveillance, recurrence rates were 32% at five years and 43% at 10 years; around one-fourth of the recurrences were adenocarcinomas [17]. Crist DW et al. in a study comparing outcomes of Whipple’s procedure done on patients with periampullary cancers over two different time periods reported a recent decline in operative morbidity and mortality [18]. Pancreaticoduodenectomy is the treatment of choice for malignant villous tumors of the duodenum, however, there is evidence of an adenoma-carcinoma-sequence and Hoyuela et al. reported adenocarcinoma to be associated in 50% cases of villous adenoma. Therefore, pancreaticoduodenectomy can be performed in selected patients of benign villous tumors with low-grade dysplasia. Mandatory postoperative endoscopic surveillance is required if local excision is performed [19-20].

## Conclusions

Tubulovillous adenomas of the duodenum are very rare with an incidence of 0.4% of all the small intestinal lesions. Although traditionally small bowel tumors are difficult to diagnose, however, a heightened index of suspicion and an increase in employment of recent diagnostic techniques such as upper gastrointestinal endoscopy and ERCP has increased the yield and decrease delays in identification. Due to the high recurrence rate of tubule-villous adenomas, a complete resection of the tumor is necessary and watchful follow-up is needed with immediate intervention in case of recurrence.
